The article "Research Progress of m6A RNA Methylation in Skin Diseases" was published in 2023. Journal: Biomed Res Int.

# Research Progress of m^6^A RNA Methylation in Skin Diseases

**DOI:** 10.1155/2023/3091204

**Published:** 2023-04-19

**Authors:** Chang Liu, Xin Wang, Shengju Yang, Shuanglin Cao

**Affiliations:** Department of Dermatology, Affiliated Hospital of Nantong University, Medical School of Nantong University, Nantong 226001, China

## Abstract

N^6^-Methyladenosine (m^6^A) is the most common mRNA modification in eukaryotes and is a dynamically reversible posttranscriptional modification. The enzymes involved in m^6^A modification mainly include methyltransferases (writers), demethylases (erasers), and methylated readers (Readers). m^6^A modification is mainly catalyzed by m^6^A methyltransferase and removed by m^6^A demethylase. The modified RNA can be specifically recognized and bound by m^6^A recognition protein. This protein complex then mediates RNA splicing, maturation, nucleation, degradation, and translation. m^6^A also alters gene expression and regulates cellular processes such as self-renewal, differentiation, invasion, and apoptosis. An increasing body of evidence indicates that the m^6^A methylation modification process is closely related to the occurrence of various skin diseases. In this review, we discuss the role of m^6^A methylation in skin development and skin diseases including psoriasis, melanoma, and cutaneous squamous cell carcinoma.

## 1. Introduction

In recent years, RNA methylation-mediated epigenetic epitranscriptome regulation has emerged as a new field of RNA biology. There are several common internal modifications of mRNA including N^6^-methyladenosine (m^6^A), N^1^-methyladenosine (m^1^A), 5-hydroxymethyl-cytosine (hm^5^C), N^7^-methylguanosine (m^7^G), and pseudouridine (*Ψ*). Among them, N^6^-methyladenosine (m^6^A) is the most frequent modification of eukaryotic mRNA with a dynamic and reversible posttranscriptional manner. The modifications of mRNA exist in the 5′ cap and 3′ poly-A regions of eukaryotes. The methylation in the 5′ untranslated region (5′UTR) of mRNA plays an important role in mRNA splicing, editing, stability, degradation, and polyadenylation, while the methylation in the 3′ untranslated region (3′UTR) contributes to mRNA outward transport, translation initiation, and mRNA structural stability maintenance with poly A-binding proteins [1]. N^6^-Methyladenosine (m^6^A) is enriched near termination codon and 3′UTR and translated near 5′UTR or in long exons [2]. Recent studies have shown that m^6^A methylation regulates cell division and proliferation, death and apoptosis in nervous system development, circadian rhythm, DNA damage response, heat shock response, and tumorigenesis in mammals [3–8]. Therefore, m^6^A methylation defect or dysregulation may disrupt gene expression to result in RNA metabolism abnormality and disease.

Recently, an increasing body of evidence indicates that the m^6^A methylation modification process is closely related to the occurrence of various dermatological diseases. In this review, we summarized the m^6^A RNA methylation and the emerging progress in skin diseases including psoriasis, melanoma, squamous cell carcinoma, Merkel cell carcinoma, and atopic dermatitis.

## 2. m^6^A Methylation

The dynamic modification of m^6^A methylation requires the participation of three types of regulators. First, m^6^A methyltransferase with the encoding gene called “Writers” catalyzes the m^6^A methylation from RNA. Second, m^6^A demethylase with the encoding gene called “Eraser” removes the m^6^A methylation in RNA. Third, m^6^A-methylated reader proteins bind to m^6^A sites in RNA to perform specific biological functions. Above enzymes play different roles of in dynamic modification of m^6^A methylation (Figure 1).

### 2.1. Writers

RNA m^6^A methyltransferases include methyltransferase-like protein 3 (METTL3), METTL5, METTL14, METTL16, Wilms' tumor 1-associated protein (WTAP), RNA-binding motif protein 15 (RBM15/15B), and zinc finger CCCH-type containing 13 (ZC3H13) [9]. The m^6^A installation of methylation is catalyzed by several methyltransferase complexes (MTC). Methyltransferase-like 3 (METTL3) is an S-adenosylmethionine- (SAM-) binding protein, which is the key methyltransferase for m^6^A methylation and the most important component of m^6^A MTC. Abnormal expression of METTL3 can change the total methylation level of m^6^A. As a structural support of METTL3, METTL14 forms a stable methyltransferase complex at a ratio of 1 : 1 to induce m^6^A RNA [10]. METTL16, as a newly discovered independent RNA methyltransferase, may be involved in the regulation of mRNA splicing and stability and binding with the METTL3/METTL14 methylation complex [11]. RBM15/15B assists in the binding of METTL3 and WTAP by directing these two proteins to specific RNA sites for m^6^A modification [12]. Other proteins, such as ZC3H13 and cofactors including WTAP, collaboratively control m^6^A methylation [13]. Taken together, these enzymes form complexes and then cooperate with each other or cofactors to regulate m^6^A methylation.

### 2.2. Erasers

Demethylase mainly includes fat mass and obesity-associated protein (FTO) and AlkB homologue 5(ALKBH5). FTO and ALKBH5 belong to *α*-ketoglutarate-dependent dioxygenase family and catalyze m^6^A demethylation in Fe (II) and *α*-ketoglutaric acid-dependent manner. They mediate the demethylation process by oxidizing m^6^A to form N^6^-hydroxymethyladenosine (hm^6^A), then converting hm^6^A to N^6^-formyladenosine (f^6^A) and finally converting f^6^A to adenosine [14]. FTO and ALKBH5 enzymes are neutral stable and can then be hydrolyzed into adenine. FTO is the first protein discovered to catalyze m^6^A demethylation and is a member of the ALKB family with a highly conserved catalytic domain. ALKBH5 was shown to be an RNA demethylase that can oxidatively reverse m^6^A modification. Unlike FTO, ALKBH5 with unique crystal structures is a specific demethylase during m^6^A RNA methylation [15]. However, at present, there are relatively few demethylases, and some other components of m^6^A methyltransferase remain to be verified. The mechanism to maintain dynamic balance with methylation and demethylation is not completely clear.

It is interesting that FTO has recently been found to preferentially target N^6^, 2′-O-dimethyladenosine (m^6^A_m_) with its major target being m^6^A_m_ in small nuclear RNAs [16]. m^6^A_m_ is found at the 5′ end of mRNA, at the first encoded nucleotide adjacent to the 7-methylguanosine cap [17]. A recent study identified a cap-specific adenosine methyltransferase (CAPAM) was responsible for N^6^-methylation of m^6^A_m_ and removed by FTO [18]. Thus, the methyltransferase to m^6^A_m_ is different from that of m^6^A.

### 2.3. Readers

Methylated reader proteins mainly include members of YTH-domain families (YTHDF1, YTHDF2, YTHDF3, YTHDC1, and YTHDC2), heterogeneous ribonucleoproteins (HNRNPC, HNRNPG, and HNRNPA2B1), and insulin-like growth factor 2 mRNA-binding proteins (IGF2BPs). There is a conservative YTH domain with the properties of single-stranded RNA-binding proteins in members of YTH-domain family. YTHDF1 facilitates the translation of m^6^A-methylated proteins by recruiting eukaryotic translation initiation factor 3 (eIF3) translation initiation complexes. YTHDF2 selectively binds to 3′UTR of m^6^A and regulates mRNA degradation to affect mRNA stability. YTHDF3 promotes protein synthesis and translation through synergetic effects with YTHDF1 to augment YTHDF2-mediated mRNA degradation [19]. YTHDF1, YTHDF2, and YTHDF3 (DF1, DF2, and DF3) and all the DF paralogs regulate the same mRNAs based on the m^6^A sites [20]. YTHDC1 is an m^6^A reader protein mediated by RNA splicing. YTHDC2 interacts with RNA helicase to provide topological regulation of translation and extension [21]. HNRNPC and HNRNPG adjust splicing and abundance of mRNA after m^6^A recognition. The phenomenon is called the “m^6^A switch” [22]. In addition, IGF2BPs identify m^6^A and enhance mRNA stability and translation in m^6^A-dependent ways [23]. These methylated reader proteins may activate downstream regulatory pathways such as RNA degradation by identifying m^6^A-modified critical sites during methylation.

## 3. Roles of m^6^A Methylation in Skin Development

Skin with rich blood vessels and a complex structure is the most easily exposed organ to the external environment. Increasing evidence demonstrates that m^6^A is closely related to skin development and regeneration. The mouse embryonic skin epithelium is initially a layer of pluripotent epithelial progenitor cells that later develop into three tissues consist of epidermis, hair follicles, and sebaceous glands. A research analyzed the potential effect of m^6^A deficiency on mouse embryonic skin epithelial progenitor by single-cell RNA sequencing and functional studies. It demonstrated that both signaling and canonical translation pathways such as Wnt signal, actin regulators, cell polarity, extracellular matrix- (ECM-) receptor interaction, and NOTCH signal were significantly downregulated after m^6^A loss [24]. Immunofluorescence imaging revealed that METTL3 deficiency in epidermal progenitor cells result in hair follicle morphology defection. After METTL3 knockout, translation initiation factors in mRNA were downregulated, while RNA metabolism and compensatory mechanisms were activated. Skin regeneration and wound repair in mammalians are maintained by epidermal progenitor cells [25, 26]. Genome editing and mouse genetics data reveal that deletion of m^6^A methyltransferase impairs the skin's ability to self-renew and heal wounds. The above findings suggested that m^6^A methylation is indispensable during skin development.

Previous studies have discovered the possible mechanism of epitranscriptome dynamics occur during epidermal differentiation. The study demonstrated that plasmacytoma variant translocation 1 (Pvt1) methylation enhanced the interaction with myelocytomatosis oncogene (MYC) and stabilized MYC protein in epidermal progenitors. It identified m^6^A methylation of Pvt1 as a key step in skin tissue homeostasis and wound repair [27]. In a recent study on skin development in goats, researchers verified 9085 m^6^A sites with differential RNA methylation in cashmere fiber growth by methylated RNA immunoprecipitation followed by high-throughput sequencing (MeRIP-seq) and RNA-seq [28]. The results proved compelling evidence that these m^6^A-modified genes were highly expressed in the skin tissue of goats. Keratins, the major components of the epithelial cytoskeleton, are responsible for maintaining the structural stability and integrity of keratinocytes, protecting cells from mechanical damage and affecting the formation of skin accessory organs. Furthermore, GO enrichment analysis showed that methylated genes were mainly involved in keratin filaments and intermediate filaments [29]. Therefore, these findings provide a theoretical basis for further research on the role of m^6^A modification in skin development and growth. It proposes a possible strategy for wound healing via regulating m^6^A modification.

## 4. Roles of m^6^A Methylation in Skin Tumors

Many studies have shown that m^6^A modification plays an important role in a variety of malignant tumors [30, 31]. The methyltransferase catalyzes the m^6^A modification on oncogenes or tumor suppressor genes. m^6^A reader proteins recognize corresponding markers through a series of biological effects, thereby to upregulate oncogene expression or downregulate tumor suppressor gene expression. On the other hand, the demethylase accelerates tumor progression via tumor-specific oncogenes [32]. These observations indicate that enhancing m^6^A modification to regulate these genes may be a novel therapeutic strategy for cancer.

Among them, one group found that FTO was upregulated while m^6^A RNA methylation was downregulated in arsenic-related human skin lesions. Moreover, FTO removal significantly inhibited arsenic-induced skin tumorigenesis [33]. Further m^6^A-seq and RNA-seq analysis revealed that neural precursor cell-expressed developmentally downregulated 4 like (NEDD4L) was the critical target of FTO during m^6^A RNA methylation, and FTO regulated NEDD4L mRNA stability via IGF2BPs. Another study revealed FTO-mediated dysregulation of mRNA m^6^A methylation as an epitranscriptomic mechanism to promote arsenic tumorigenesis. Analysis of gene expression profiles showed higher expressions of m^6^A effectors, especially METTL3, in arsenic-exposed groups than low-arsenic-exposed populations. Further experiments found that arsenic promoted m^6^A methylation by up-regulating METTL3 to increase the secretion of inflammatory factors including interleukin- (IL-) 6, IL-17, and IL-10 in human keratinocytes. Keratin 1 (KRT1) and keratin 10 (KRT10) reflecting skin injury were also significantly increased [34]. Another study demonstrated that METTL14 facilitated global genome repair (GGR) by regulating m^6^A RNA methylation-mediated DNA damage-binding protein 2 (DDB2) translation and inhibits ultraviolet B- (UVB-) induced skin tumorigenesis. METTL14 knockout suppressed m^6^A RNA methylation and translation in transcripts of DDB2 [35]. Therefore, METTL14 is an important specific autophagy target to regulate GGR and attenuate UVB-induced skin tumorgenesis.

### 4.1. Melanoma

Melanoma is a serious and life-threatening skin malignancy [36]. About 75% of patients suffering skin tumor die of melanoma. Several m^6^A regulators including METTL3, YTHDF1, HNRNPA2B1, FTO, and IGF2BP3 are involved in melanoma (Figure 2). Studies have shown that the expression of METTL3 is upregulated in human melanoma cell lines, and it promotes melanoma cell proliferation. Further research suggested METTL3 accelerated invasion and migration of melanoma cells by upregulating matrix metallopeptidase 2 (MMP2) [37]. In addition, the growth speed of YTHDF1-deficient melanoma cells was lower than that of wild type (WT) cells in mice. Moreover, the control rate of melanoma by immunotherapy in YTHDF1 knockout mice increased to nearly 100%, while the rate was only 40% in WT mice [38]. FTO was the first found RNA m^6^A demethylase among the m^6^A regulators. Studies have shown that FTO stimulates melanoma growth. FTO knockout increased m^6^A methylation of genes including PD-1 (programmed cell death protein 1), CXCR4 (C-X-C motif chemokine receptor), and SOX10 (Sry-related HMG-box-10) in melanoma cells and thereby enhanced the susceptibility to interferon therapy [39]. METTL3 could modulate the mRNA level of uridine cytidine kinase 2 (UCK2) through m^6^A modification to enhance its stability in melanoma. In addition, UCK2 enhanced the migration and invasion ability of melanoma cells by activating the Wnt/*β*-catenin pathway [40]. Both YTHDF1 and HNRNPA2B1 were upregulated in melanoma. The diagnosis sensitivity for melanoma with these two gene-combined screening increased approximately 10% compared to single-gene screening. The expression of p53 and associated genes including cyclin-dependent kinase 1 (CDK1) and CDK2 was positively correlated with upregulation of YTHDF1 or HNRNPA2B1 [41]. A three-gene prognostic marker including IGF2BP3, RBM15B, and METTL16 was constructed by analyzing the differently expression of m^6^A regulatory factors in tumor samples and normal samples. It was demonstrated that IGF2BP3 promoted proliferation and migration of melanoma cells *in vitro.* The expression of IGF2BP3 was positively correlated with lymph node metastasis and immune cells infiltrating [42]. These results provided potential targets of novel drugs for melanoma.

Some researchers analyzed the gene expression profiles, copy number variation (CNV), and single-nucleotide polymorphism (SNP) data from The Cancer Genome Atlas (TCGA) databases. The study showed that 15 genes were changed on mRNA expression and m^6^A regulatory proteins such as RBM15, YTHDF1, WTAP, and METTL14 genes in melanoma with a higher degree of genomic variation and a worse prognosis. Then, they identified a subset of molecules with immunological effects based on m^6^A regulatory proteins [43]. The study provided a new and effective strategy for the treatment of cutaneous melanoma. The above results suggested that the regulatory proteins of m^6^A methylation, including methylation on writing proteins, methylation reading proteins, and demethylases such as METTL3, YTHDF1, and FTO, play an important role in the development of melanoma. It provides a reliable theoretical basis for the treatment of melanoma and the development of drugs.

### 4.2. Cutaneous Squamous Cell Carcinoma

Cutaneous squamous cell carcinoma (cSCC) is the second most common skin malignancy, accounting for 20% of nonmelanoma skin cancers. The most important physical factor causing the incidence of cSCC is sunlight ultraviolet rays especially UVB. Excessive sunlight exposure could lead to cell mutation and tumorgenesis. Studies have shown that exposure to UVB and arsenic resulted in upregulation of m^6^A-binding protein YTHDF1 expression in skin keratinocytes, even skin mutation and oncogenesis to cause cSCC [44].

The m^6^A methyltransferase METTL3 is also a key gene to regulate the occurrence of cSCC genesis. METTL3 was upregulated in cSCC, and METTL3 knockout disrupted the characteristics of stem cells in cSCC. METTL3 deficiency decreased colony-forming ability and suppressed tumorigenicity *in vivo* by reducing m^6^A levels and *Δ*Np63 expression in cSCC. Exogenous *Δ*Np63 overexpression partially restored the proliferation of METTL3-knockout cSCC cells [45].

m^6^A RNA methylation in cSCC was not studied as extensively as other related squamous cell carcinomas such as oral squamous cell carcinoma (OSCC), hepatocellular carcinoma (HCC), and gastric cancer (GC). Studies have shown that METTL3 promoted *BMI1* translation in OSCC under the cooperation with m^6^A reader IGF2BP1 and promoted OSCC proliferation and metastasis [46]. Combination of YTHDF1 silencing and epidermal factor growth receptor (EGFR) inhibition synergically suppressed the malignancies of HCC cells [47]. The expression profile variation of YTHDF1 was significantly associated with the high-risk subtype of GC patients, suggesting that YTHDF1 might be a potential target in GC early diagnosis [48]. These studies verified the detailed mechanism of m^6^A methylation in cutaneous squamous cell carcinoma.

### 4.3. Merkel Cell Carcinoma (MCC)

MCC is a highly aggressive and rare skin cancer [49]. Merkel cell polyomavirus (MCPyV or MCV) can be detected in 80% of cases with MCC [50]. MCPyV is related to the animal tumor virus simian virus 40 (SV40). The differential splicing of the mRNA sequence produces the oncoprotein T antigen, which encodes the large T, small T, and 57 kT antigens [51]. One group used genomic screening of copy number aberrations along with transcriptomic analysis to investigate regions with amplification that harbor differentially expressed genes. They found that YTHDF1 was highly amplified and expressed in Merkel cell lines. YTHDF1 activated cap-dependent translation. Then, the translation initiation factors eIF3A and eIF3B cooperated synergistically, leading to high tumorigenicity. Moreover, YTHDF1 knockdown inhibited eIF3 to attenuate proliferative and clonal capacity. Survival data analysis showed that MCC patients with more YTHDF1 expression had lower overall survival compared with those with less YTHDF1. In other words, YTHDF1 level was negatively correlated with MCC patient prognosis and overall survival. Furthermore, the study identified m^6^A modifications on small T antigen mRNAs [52]. The study suggested a possible relationship between YTHDF1 amplification and MCPyV gene expression. YTHDF1 could be a novel prognostic marker for MCC.

In summary, m^6^A-binding protein FTO, METTL3, METTL14, and YTHDF1 expression were involved in skin lesion and oncogenesis. FTO promotes oncogenesis via IGF2BPs. METTL3 increases inflammatory factor secretion in human keratinocytes and enhanced *Δ*Np63 expression in cSCC. METTL14 facilitates GGR to suppress UVB-induced skin tumorigenesis. YTHDF1 activates translation initiation factors to high tumorigenicity in MCC (Figure 3).

## 5. Roles of m^6^A Modification in Inflammatory Skin Diseases

### 5.1. Psoriasis

Psoriasis is a common, complex, and chronic inflammatory disease that severely reduces patients' quality of life. The hallmark of psoriasis is uncontrolled proliferation and differentiation of keratinocytes by persistent inflammation. Previous studies have shown that methylated transcripts were mainly related to the Wnt signaling pathway in skin lesions of psoriasis patients. The Wnt gene family encodes a group of highly conserved secretory signal proteins involved in cell differentiation, proliferation, and immune-mediated inflammatory responses [53–55]. It is noted that m^6^A methylation regulated these key pathogenic processes including dendritic cell (DC) activation in psoriasis by altering Wnt gene expressions [56, 57]. Tumor necrosis factor- (TNF-) *α*/IL-23/Th17 axis is regarded as a key factor in inflammation exacerbation and lesion aggravation in psoriasis, being critical for the expansion of inflammation and aggravation of skin lesions in psoriasis vulgaris [58]. One study detected m^6^A methylation in psoriasis patients by MeRIP-Seq and RNA-Seq. The results showed that IL-17A and TNF-*α*, as two key genes of the TNF-*α*/IL-23/Th17 axis, are upregulated m^6^A methylation in skin lesions of psoriasis patients [59].

Additionally, the mRNA and protein levels of m^6^A writer WTAP were significantly increased in psoriasis patients especially in the epidermis. Overexpression of WTAP promoted the proliferation of keratinocytes, which may be possibly related to the upregulation of cyclinA2 and CDK2 [60]. The above findings suggest that m^6^A may be an important trans-epigenetic modifier to regulate proliferation, differentiation, and inflammation of psoriatic keratinocytes.

### 5.2. Atopic Dermatitis (AD)

AD is a common and chronic inflammatory skin disease affecting approximately 10-25% of children and 7-10% of adults. It is characterized by disturbances in epidermal structure and keratinocyte differentiation, as well as excessive T cell-mediated inflammation with a complex genetic condition [61]. The pathogenesis is related to mutations in genes encoding epidermal structural proteins, barrier enzymes, and their inhibitors. Recent studies demonstrated a critical role of epigenetic changes in AD [62]. One study demonstrated that circRNAs regulated macrophage-mediated inflammation via analyzing differential expression profile of circRNAs by circRNA microarray. Further results also showed that Hsa_circ_0004287 reduced the stability of MALAT1 by competitively binding to IGF2BP3 and MALAT1 in an m^6^A-dependent manner in 2,4-dinitrochlorobenzene- (DNCB-) induced dermatitis. Low levels of MALAT1 promoted ubiquitinated degradation of S100A8/S100A9, thereby prevented p38/mitogen-activated protein kinase phosphorylation and macrophage-mediated inflammation, and finally inhibited M1 macrophage activation [63]. The existing studies on m^6^A RNA methylation in atopic dermatitis proposed a possible role of macrophage-mediated inflammation in disease progression.

## 6. Roles of m^6^A Modification in Other Skin Diseases

Scleroderma is an autoimmune connective tissue characterized by organ fibrosis, immune abnormalities, and vascular damage [64]. Although scleroderma is a rare disease with a low prevalence and incidence, it has a high mortality rate [65]. A recent study identified m^6^A-tagged mRNAs in a mouse model of bleomycin-induced scleroderma by m^6^A supratranscriptomic microarrays and m^6^A RNA immunoprecipitation qPCR. The results showed that there were differences in the m^6^A methylation of 843 mRNAs and include the methylation and the expression of Hras, Saa1, Ccl3, Ccl9, and Il1b [66]. This study revealed the involvement of m^6^A methylation in scleroderma.

Cutaneous T-cell lymphomas (CTCL) are a rare type of non-Hodgkin lymphoma characterized by cutaneous infiltration of malignant lymphocytes [67]. Recent studies have uncovered a role for METTL3-mediated m^6^A modification in CTCL progression. The results showed that METTL3 significantly downregulated CTCL cells both *in vivo* and *in vitro*. Furthermore, METTL3 small interfering RNAs and RIP assay indicated that cyclin-dependent kinase inhibitor 2A (CDKN2A) was a key regulator in CTCL, and insufficient methylation blocked the interaction between CDKN2A and m^6^A reader IGF2BP2, resulting in mRNA degradation [68]. This is the first study to describe the role of m^6^A in CTCL development and provide a potential biological target for therapy.

Sequestosome 1 (SQSTM1) is a vital protein marker serving as a selective autophagy receptor [69]. SQSTM1/p62 was significantly downregulated in the epidermis of diabetic patients and in the db/db mouse model with chronic hyperglycemia. Knockdown of SQSTM1 led to the impairment of autophagic flux. In addition, the m^6^A reader protein YTHDC1 interacting with SQSTM1 mRNA was attenuated in keratinocytes during hyperglycemia. *In vivo*, knockout of endogenous YTHDC1 or SQSTM1 suppressed epidermal autophagy and impaired the biological functions of keratinocytes including promoted apoptosis and delayed wound healing. The results showed that YTHDC1 interacted with ELAV-like RNA-binding protein 1/HuR (ELAVL1) and cooperatively regulated the expression of SQSTM1 [70]. This study reveals that YTHDC1 regulated autophagy by regulating the stability of SQSTM1 nuclear mRNA in diabetic keratinocytes.

One group described m^6^A modification patterns in hyperplasia scars (HS) and normal skin (NS) tissues by m^6^A sequencing and RNA sequencing. Several targets of m^6^A-associated RNA were immunoprecipitated and verified by real-time quantitative PCR. The results showed that 14791 new m^6^A peaks appeared in the HS samples, while 7835 peaks disappeared. It suggested that the m^6^A-related genes in HS are associated with fibrosis-related pathways. In addition, they identified differentially expressed mRNA transcripts in HS samples with hypermethylated or hypomethylated m^6^A peaks [71]. This study maps the m^6^A epitranscriptome of human HS, which may help to elucidate the possible mechanisms of m^6^A-mediated regulation of gene expression.

## 7. Limitations and Challenges of Current Research on m^6^A Methylation

There is no study to exactly confirm the specific mechanism in dynamic m^6^A regulation in skin disease. Only a few studies were published on the mechanisms that control the expressions and activities of m^6^A “Writers,” “Erasers,” and “Readers” in the skin, especially the “reader.” Previous studies have confirmed that m^6^A methylase has dual effects of cancer promoting or suppressing. METTL3 serves as an apoptosis driver in high glucose-reliant human lens epithelial cells (HLEC), while WTAP acts as an inhibitor in human natural killer/T cell lymphoma (NKTCL) cell lines [13, 27]. This study demonstrates the existence of a two-way regulatory mechanism for methylation. Therefore, the research on the roles of m^6^A methylation in skin tumors and skin inflammatory diseases still needs to be further explored.

The total amount of m^6^A in RNA can be probed by several methods, including two-dimensional thin layer chromatography [72], m^6^A dot-blot [73], and HPLC-MS/MS (high-performance liquid chromatography-tandem mass spectrometry) [74]. However, these approaches are not suitable for high throughput identification and localization of modified sites. MeRIP-seq, also known as m^6^A-seq (m^6^A RNA immunoprecipitation sequencing), relies on RNA fragmentation but incapable of single-nucleotide resolution detection in methylation sites [75]. Although various methods have been found currently, there are still so many challenges and difficulties to detect m^6^A methylation. Some more effective methods especially in the skin are urgently needed.

There are already some drugs targeting methylations. The nonsteroidal anti-inflammatory agent meclofenamic (MA) has a strong inhibitory effect on FTO and is expected to become a demethylase inhibitor. MA2, an ethylester derivative of MA is hydrolyzed inside the cell to its active form MA. MA2 increased m^6^A methylation in HeLa cells and had better cellular permeability than MA [76, 77]. However, these drugs have not been tested in clinic for their effectiveness. It is well-known that immunotherapy plays a significant role in the treatment of skin diseases such as melanoma. Various studies have confirmed that m^6^A methylation regulates innate immune response [56, 77]. It was demonstrated that m^6^A methylation was a crucial regulator of T cell homeostasis. T cells carrying m^6^A modifying agents may be an effective target for the treatment of autoimmune diseases [78]. These studies showed the potential application of this mechanism in immunotherapy. Although they can provide potential pharmacological targets, the clinical effects should be further verified.

## 8. Conclusions

Taken together, m^6^A is dynamically regulated in many physiological and pathological processes of dermatological diseases. RNA methylation is regulated by methylase, demethylase, and methylation reader proteins, and the process is reversible. RNA methylation is a relatively new field. In recent years, m^6^A has been prominently discovered in various skin diseases. However, many unknowns still exist in the epitranscriptome modification of RNA. The detection method of m^6^A methylation needs improvement. The efficacy of methylation-modifying agents needs further clinical studies. Epitranscriptome modification has attracted more and more attention in regulating immune response and immunotherapy. Exploring key epitranscriptome variation sites and developing corresponding immunotherapy drugs have become research hotspots and have good development prospects.

## Figures and Tables

**Figure 1:** The types and roles of enzymes in dynamic modification of m^6^A methylation. The m^6^A RNA methylation is dynamically regulated by writers, erasers, and readers to add, remove, or recognize m^6^A, respectively. Writers include METTL3, METTL5, METTL14, METTL16, WTAP, RBM15/15B, and ZC3H13. Erasers, FTO and ALKBH5, are two known demethylases. Readers are proteins that recognize the m^6^A sites and perform multiple functions in nucleus or cytoplasm, including YTHDF1, YTHDF2, YTHDF3, YTHDC1, YTHDC2, HNRNPC, HNRNPG, and IGF2BPs. These enzymes are involved in RNA splicing, translation, structure switching, and RNA decay during m^6^A RNA methylation.

**Figure 2:** Mechanistic illustrations of the regulatory and functional roles of m^6^A in melanoma. Several m^6^A regulators including METTL3, YTHDF1, HNRNPA2B1, FTO, and IGF2BP3 are involved in melanoma. METTL3 increases mRNA level of UCK2 through m^6^A methylation to enhance its stability in melanoma. Then, UCK2 promotes the migration and invasion ability of melanoma cells by activating the Wnt/*β*-catenin pathway. METTL3 also accelerates invasion and migration of melanoma cells by elevating MMP2 expression. In addition, YTHDF1 or HNRNPA2B1 promotes p53 signal pathway via m^6^A methylation to tumorgenesis. FTO reduces m^6^A methylation to inhibit gene expressions including PD-1, CXCR4, and SOX10 but stimulate melanoma growth in melanoma cells. IGF2BP3 promotes proliferation and migration of melanoma cells.

**Figure 3:** Process of m^6^A methylation induced by UVB and arsenic in skin. Several m^6^A regulators, including methylation on writing protein METTL3, methylation reading protein YTHDF1, and demethylase FTO, play an important role in the development of melanoma, even skin mutation and canceration to causing cSCC especially after UVB and arsenic exposure. FTO regulates NEDD4L mRNA stability to promote skin neoplasms via IGF2BPs. METTL3 increases inflammatory factor secretion including IL-6, IL-17, and IL-10 in human keratinocytes; then, KRT1 and KRT10 reflecting skin injury are also significantly elevated. METTL3 also enhanced *Δ*Np63 expression in cSCC. METTL14 facilitates GGR to suppress UVB-induced skin tumorigenesis. YTHDF1 activates cap-dependent translation. Then, the translation initiation factors eIF3A and eIF3B cooperate synergistically to possibly lead to high tumorigenicity in MCC.

## Data Availability

All data are available on request.
